The article "Analysis of Metabonomic Characteristics after Exercise Fatigue Based on NMR" was retracted in 2023. Reasons: signs of a paper mill; suspected computer-generated content; unreliable results or conclusions; lack of ethics approval or compliance.

# Analysis of Metabonomic Characteristics after Exercise Fatigue Based on NMR

**DOI:** 10.1155/2022/9041293

**Published:** 2022-08-13

**Authors:** YuRong Chen, Xiaoqiang Wang

**Affiliations:** Hainan Medical University, Haikou, Hainan 571199, China

## Abstract

In order to better understand the changes of body metabolism of athletes before and after exercise, this paper proposes a method of metabonomics feature analysis after exercise fatigue based on NMR. This paper makes a retrospective analysis on the metabonomic characteristics of urine of middle and long distance runners after 30 minutes of a heavy load training class based on NMR. The experiment analyzes the urine of athletes by combining NMR technology and metabonomics principle. The experimental results show that the Q2 value of this experiment is greater than that of all comparisons, and r2x and r2y are 0.436 and 0.85, respectively. *Conclusion*. This method can effectively analyze the changes of body metabolism after athletes' fatigue, so as to better alleviate athletes' fatigue after exercise.

## 1. Introduction

Training and competition is an important part of competitive sports. Its purpose is to continuously tap the sports potential of the human body, maximize the competitive ability of athletes, and create excellent sports results [1]. “Faster, higher, and stronger” is one of the tenets of the modern Olympic spirit. In competitive sports, the competition is becoming more and more intense, and the intensity of competition and training is also approaching the limits of the human body. These will inevitably bring varying degrees of decline to the body's functional state. The challenge of how to quickly restore the functional state and ensure the continuity and efficiency of training and competition has always been the goal pursued by the majority of coaches and athletes.

Exercise causes changes or adaptations of body material and energy metabolism, which must be reflected in metabolites [2]. Metabonomics is a discipline developed in the late 1990s. It is a system biology discipline that has developed rapidly since the human genome project, with high-throughput detection and data processing as the means, information modeling and system integration as the goal, and group index analysis as the basis [3–5]. Metabonomics reflects the relationship between the collection of molecules and their functions by measuring the changes in the concentration and proportion of various metabolites in the body and objectively reflects the characteristics of the overall changes of the organism. Metabonomics research is not limited to the details of the changes of a substance or metabolic pathway after the body is affected by various external conditions, but focuses on the overall changes of metabolites after a series of changes. Different from any previous detection method using a single or one aspect of indicators, metabonomics research can more accurately and comprehensively reflect the overall and dynamic changes of the body state [6].

Nuclear magnetic resonance (NMR) is a physical phenomenon of the interaction between alternating magnetic field and matter, which was first confirmed by experiments in 1946 [7]. The discovery of nuclear magnetic resonance (NMR) is of great significance. It not only provides direct verification for the basic principles of quantum mechanics but also provides an indispensable means of analysis and measurement for the research in many disciplines.

In order to better investigate the physical condition of athletes after sports fatigue, the application of NMR technology to the analysis of metabonomics after sports fatigue can better analyze it, so as to better make athletes get timely adjustment.

## 2. Literature Review

Nuclear magnetic resonance technology mainly has two subject branches: nuclear magnetic resonance spectroscopy and magnetic resonance imaging (MRI) [8, 9]. Nuclear magnetic resonance spectroscopy is developed based on the chemical shift theory, which is mainly used to determine the chemical composition and molecular structure of substances. Nuclear magnetic resonance imaging technology was born in 1973. It is a nondestructive measurement technology, which can be used to obtain the internal structure images of a variety of substances. Due to the abundant information that NMR can obtain, it is widely used in many fields, such as analytical chemistry, life science, material detection, oil exploration, and water resources exploration.

Metabolomics (metabolomics/metabonomics) is the process of studying a series of changes in the type, quantity, and even the functional state of an organism after it is disturbed (such as gene changes or environmental changes) and its endogenous metabolic substances are stimulated. Metabonomics usually regards biology as a whole and focuses on exploring the relationship between internal organs, tissues, and endogenous substances. At the same time, it can also show a series of biological events that occur in the physiological activities of its body under the influence of external and internal factors [10]. Since the 1980s, metabonomics has begun to sprout. In 1985, Yang B. analyzed the urine of rats through NMR technology. Compared with previous measurements, the metabolites measured in this experiment were more diverse and comprehensive, which made them realize that this may be a major breakthrough in systems biology. At the same time, after years of research, the concept of metabonomics was formally put forward in 1999 [11]. Its metabolome usually refers to a tissue, organ or cell and the collection of all metabolic components, generally refers to some small molecular substances. The so-called metabonomics is a subject that studies the corresponding changes of some substances in the body caused by the metabolism of organisms. Therefore, metabonomics helps to analyze the essence of metabolism of life activities as a whole [12].

Systems biology research based on omics technology mainly covers genomics, proteomics, metabonomics, transcriptomics, and so on [13–16]. Among them, the contents of each omics are different. For example, genomics mainly studies the genome structure of biological systems, including the functions of its fund groups and the products they express. Proteomics focuses on the study of protein characteristics of biological systems on a large scale. The main research content of metabonomics is to study the changes of all endogenous substances in the body under the stimulation of the external environment. In essence, metabonomics can be considered as a further in-depth study of the first two omics. With the continuous development of omics technology, people have gradually deepened their understanding of it. More and more scholars have realized that because many genes are recessive genes, sometimes changes in their genomes do not necessarily show up, so sometimes, their physical functions are not affected. Although the protein content in the body will change correspondingly due to the stimulation of the external environment, the protein itself may not have activity, so it is also difficult to have some significant effects on the body. In addition, due to the compensation effect, the deletion of some proteins or genes will be compensated by the relevant proteins and genes in the body, and eventually will not cause symptoms. However, the change of some small molecular substances is the result of this series of symptoms. These small molecular substances can intuitively, accurately, and comprehensively reflect the physiological status of the organism.

Metabolome is usually between tissues, cells, proteins, and genes. It is generally in the midstream of biological information flow. It plays a connecting role in the process of information transmission. Metabolism is the most basic feature of an organism, and the life activities of organisms and cells are more shown in their metabolism [17]. These include hormones, receptors, cell communication, and neurotransmitters. Therefore, metabonomics of organisms is considered as the terminal of omics research [18]. Compared with proteomics and genomics, metabonomics can more intuitively reflect the state of tissues, cells, and organs in the body, including the impact of external drugs, stimuli, and nutrition [19]. The following is the flow chart of metabonomics experimental research as shown in Figure 1.

Based on the abovementioned research, this paper proposes a method of omics metabolism research after exercise fatigue based on NMR. In this method, the metabonomics method is used to analyze the urine of athletes after exercise by using NMR technology. The urine is analyzed to obtain various physical indicators of athletes before and after exercise, to analyze the physical impact on athletes after exercise, and then to formulate effective measures to alleviate the exercise fatigue of sports mobilization.

## 3. Research Methods

### 3.1. Basic Principles of Nuclear Magnetic Resonance

Nuclear magnetic resonance (NMR) refers to the phenomenon of nuclear resonance transition between energy levels under the action of an external magnetic field. The magnitude of nuclear magnetism is generally expressed by the magnetic moment *µ*, *µ* is directional, *μ*=vhI, *h* is Planck constant, and I is the spin quantum number, which is referred to as spin for short. The spin magnetic ratio *v* is actually a measure of the size of the nuclear magnetism. A large value of *v* means that the nuclear magnetism is strong and vice versa. Among natural isotopes, the *v* value of hydrogen nuclei (protons) is the largest (42.6 MHz/T), so the detection sensitivity is the highest, which is one of the important reasons why protons were first selected as NMR research objects.

When a nucleus with magnetic moment (*I* ≠ 0) is placed in a magnetic field, the behavior of the nucleus in the magnetic field is like the motion of a gyroscope—Larmor precession, and its frequency is determined by formula (1):

(1) $$\begin{array}{c} \omega =2\pi v, \end{array}$$

where *ω* is the angular frequency and *v* is the Larmor precession frequency. When the frequency of the external RF field is equal to the Larmor frequency of the atomic nucleus, the nucleus in the low-energy state will absorb the RF energy and transition from the low-energy state to the high-energy state, which is the phenomenon of nuclear magnetic resonance. Nuclei without a spin (*i* = 0) have no magnetic moment, and NMR signals cannot be observed in such nuclei, such as  ^14^*C*,  ^16^*O*,  ^32^ *S*, etc.; nuclei with *i* = 1/2 are the most studied nuclei in NMR, such as  ^1^*H*,  ^13^*C*,  ^19^ *F*,  ^15^ *N*, etc.

### 3.2. Study on the Metabolomic Characteristics of Urine of Middle and Long Distance Runners after 30 Minutes of Heavy Load Training Based on NMR

#### 3.2.1. Research Subjects

In this paper, the subjects of the study on the metabolomic characteristics of urine of middle and long distance runners after 30 minutes of heavy load training class based on NMR were retrospectively analyzed. Fourteen male athletes in the middle and long distance running groups of a city track and field team were selected as the research subjects. The average age of the athletes was 17.33 ± 1.58 years old, the height was 173.84 ± 3.04 cm, the weight was 57.57 ± 4.33 kg, the body mass index (BMI) was 17.98 ± 0.73, the fat index (FBF) was 11.24 ± 1.23, and the maximum oxygen uptake was 66.06 ± 2.98. Among them, there are 5 elite athletes, 6 first-class athletes, and 3 second-class athletes.

#### 3.2.2. Training Course Contents

Time: on the morning of December 14, 2013 (Saturday)

Special endurance: 8000 m running; average 85 s/cycle (400 m); the total time is 28 min 20 s. The last 5 laps should be kept at 90-86-84-82-78 (s), and rest for 20 min.

Special speed endurance: (500 m fast running +100 m jogging) x16 times. They were divided into two groups (12 + 4): the first 12 times were a group (running with ordinary sneakers) and the last 4 times were a group (running with spikes). The interval between the two groups was 6 min. The intensity of the first group was 87-85-84-82-80s (about 500 m fast running). Intensity of the second group: 80-78-75-72s (about 500 fast running time).

The training course is in the late stage of the preparation period of the annual training plan. The main task of this stage is to improve the special ability. On the basis of aerobic ability, we develop anaerobic ability and mainly improve the mixed energy supply ability of phosphate system, glycolysis system, and aerobic oxidation system. As the athletes live together and eat in the same canteen, it is easy to achieve a unified work and rest time and the same diet.

Urine samples were taken before and 30 min after training (Figure 2). This experiment was approved by the experimental ethics committee. All athletes understand the purpose of this experiment, agree to carry out the experiment, and comply with the requirements of the experiment schedule, diet, etc.

In order to determine the load intensity and load of the competition, this study detected the heart rate during exercise (polars610i telemetry heart rate meter, Finland) and athletes' subjective physical feeling scale (RPE) (using the method of questionnaire survey by researchers).

#### 3.2.3. Sample Collection and NMR Spectrum Collection

In this paper, the sample collection and NMR spectrum collection were analyzed retrospectively. Urine samples with a volume of 500 were collected in EP tubes containing 20 *μ*L1%(*w*, *v*)NaN_3_ and stored in refrigerators at −80°C. Before NMR spectrum collection, we add phosphate heavy water buffer solution (1.5 M, PH7.4, containing 2.26 mM sodium 2,2,3,3-tetradeuterate-3-trimethylsilybutyrate (TSP)) to control the pH value of the sample within a small range. After centrifugation (12000 g, 4°C, 10 min), we take supernatant (500 *μ*L) and transfer it to a 5mmnmr test tube, D2O lock field, TSP calibration (*δ*0.00).

When collecting the  ^1^*H* NMR spectra of urine samples, the NoesyPrld pulse sequence of pre saturated water peak (RD-90 °-t1-90 °-tm-90 °-ACQ) was used. When mixing, TM was 120 ms, and T1 between the first two 90° pulses was 6.6 *μ*s. The other parameters are the same as the one-dimensional NMR spectra of the water-soluble extracts. 128 FI, D64k data points, 20.4 ppm spectral width, 2.66 s acquisition time (ACQ), and water peak suppression is completed within 4S of the cycle delay (RD).

Two-dimensional presaturated water peak pulse gradient field  ^1^*H*- ^1^*H* correlation (COSY) and two dimensional  ^1^*H*- ^1^*H* total correlation (TOCSY) with a water gate were randomly collected from some samples to confirm the spectral peak assignment of one-dimensional hydrogen spectrum. All NMR experiments were carried out on a 600 MHz broker AvanceIIIHD NMR spectrometer with an ultralow temperature probe at 298 K.

#### 3.2.4. Multivariate Statistical Analysis

In order to mine the metabolite information in one-dimensional  ^1^*H* NMR spectra, a series of processing were carried out for all one-dimensional  ^1^*H* NMR spectra: (1) one-dimensional  ^1^*H* NMR spectra were multiplied by a 0.3 Hz broadened window function before Fourier transform, (2) Fourier transform, (3) manual phase modulation, (4) baseline correction; (5) reference TSP (*δ*0.00) calibration (6) perform peak alignment carefully, and (7) the  ^1^*H* NMR spectra of urine were divided into 3000 integration sections with a width of 0.003 ppm. The abovementioned operations were carried out in the software Mestrenovav8.1.4 (mestrelab research.l), (8) remove the integral position of *δ*5.20∼4.70 water peak and the wide peak signal of *δ*6.00∼5.20 urea from all spectral integration data, (9) normalize the remaining integral data to eliminate the concentration difference between samples, 10) the normalized data are input into SIMCA-P + 12.0 (Umetrics, Umea, Sweden) software package for centralized and scaled processing, 11) principal component analysis (PCA), least square discriminant analysis (PLS-DA) and orthogonal least square discriminant analysis (OPLS-DA) were performed. PCA and PLS-DA score charts are displayed by the first and second principal components, and OPLS-DA score charts are displayed by the first predictive principal component and one orthogonal component [20].

According to OPLS-DA model, the VIP (the importance of variables in mapping) value of variables is extracted, and the variables with VIP >1 are regarded as the metabolites with potential contribution to grouping.

We calculate the correlation coefficient (*R*) between variables and predicted principal components in Java environment and determine the variables with significant correlation according to the critical value standard when *R* is greater than *P*=0.05. This variable has a significant statistical significance for grouping. To determine the critical value, we first calculate the degree of freedom d*f* according to the formula d*f*=*n*_1_+*n*_2_ − 2, where *n*_1_ and *n*_2_ are the respective sample numbers of two groups in the OPLS-DA model, and then query the critical value of the correlation coefficient when *P*=0.05 in the correlation coefficient boundary value table according to the F value. To sum up, there are two criteria for selecting variables that contribute to the grouping in this study: VIP >1 and |*r*| > *r* (critical value *P*=0.05). The OPLS-DA load graph is used to determine which metabolites contribute to the grouping. The significance of the difference in metabolite concentration between groups is determined by calculating the absolute value |*r*| of the correlation coefficient. This value is greater than the *R* critical value of *P*=0.05, but less than the *r* critical value of *P*=0.01, and the color on the map is yellow. This value is greater than the *r* critical value of *P*=0.01, and the color on the load diagram is red. If the value is less than the *R* critical value of *P*=0.05, the color is blue. R2X(cum), R2Y()cum, and Q2 (cum) are used to test the robustness of PCA, PLS-DA, and OPLS-DA models. The larger these parameters are, the more reliable the model is. The intercept of Q2 regression curve in the arrangement experiment diagram is negative and all Q2 values on the left are lower than those on the right, indicating that there is no over fitting phenomenon [21].

### 3.3. Energy Metabolism Pathway

#### 3.3.1. Raw Phosphoric Acid System

Creatinine is a metabolite of the human phosphagen system (creatine phosphate or creatine). In this experiment, the content of creatinine in urine of athletes in the middle period of training was significantly higher than that at the beginning of training (more than 30%), and gradually fell back at the end of training. Compared with that at the beginning of training, there was no significant change, indicating that the metabolism of the pro-phosphate system showed a trend of rise first and then decline in this heavy load training stage. As shown in Figure 3, the production of creatinine mainly depends on two ways: first, creatine phosphate removes 1 molecule of water and phosphoric acid to produce creatinine. In addition, creatine can be directly dehydrated into creatinine. As the fastest source of ATP biosynthesis in vivo, creatine phosphate and creatine also play an important role in the internal and external transport of mitochondria. The creatine pool of the human body is mainly composed of two, which is an important source of energy storage and utilization of the body, and reflects the ability of the body to quickly supply energy. In addition, some scholars have found that there is a positive correlation between the content of urinary creatinine and the functional state of athletes' muscles. The increase of the content is the performance of the improvement of muscle function. Therefore, urinary creatinine is often used as an important indicator to evaluate the functional state of athletes.

#### 3.3.2. Glycolysis System

Lactic acid is the product of energy supply from the decomposition of glucose in the anaerobic state. Compared with the beginning of the training, the lactic acid content in the urine of the athletes at the middle and end of the training at this stage has significantly increased, indicating that the glycolysis energy supply is very strong at this training stage.

Sugar is the most important energy source in the process of human movement. Long time training and competition result in a large amount of output, decomposition, and utilization of glycogen (liver glycogen and muscle glycogen) in the body. Although the human body can continue to synthesize glucose through gluconeogenesis, it cannot meet the needs of training and competition under heavy load. At this time, glucose is required to decompose under anaerobic conditions for energy supply, that is, glycolysis for energy supply. As shown in Figure 4, glycolysis is a process of decomposing into lactic acid without oxygen and providing energy at the same time. In this process, each molecule of glucose decomposed can produce 2 molecules of pyruvate and 2 molecules of ATP. Since the fermentation process is mainly completed in the cytoplasm, no oxygen is required. In the anoxic state, pyruvate can also be reduced to lactic acid by the action of lactate dehydrogenase and hydrogen. Therefore, the human body may cause the increase of lactic acid under the conditions of hypoxia and oxidative stress.

## 4. Results and Discussion

The experimental results were analyzed retrospectively. See Table 1 for the changes of athletes' heart rate. We conduct NMR spectrum analysis on the collected urine samples to observe the differences in metabolic patterns of middle and long-distance runners before and after heavy load training.

In terms of the total training volume, the training volume in the third week is the peak of the training stage, reaching 186480 m. In the third week, the training volume of general endurance and speed exercises reached 13000 m and 3080 m, respectively, reaching the maximum in the same quality exercises at this stage. In terms of special endurance, from the second week, it increased by 26000 m compared with the first week, and changed little in the next three weeks of training. In the first week of training, the proportion of general endurance training was the largest, reaching 77.1%, and the proportions of speed endurance, special endurance, special speed endurance, and speed training were 7.2%, 5.7%, 8.5%, and 1.5%, respectively. In the second week, the proportion of various quality training has changed. In particular, the amount of special endurance training has increased by 26000 m, reaching 21.0%. The amount of other quality training has basically remained unchanged. From the change trend in Figure 5, the increase of special endurance training in the last 3 weeks is the most obvious.

In this study, there is cluster distribution between PCA, PLA-DA, and OPLS-DA sample scores. The Q2 value of the OPLS-DA model is 0.771, greater than 0.4. The arrangement experiment shows that the Q2 value on the far right is greater than that on all the left and R2X and R2Y are 0.945 and 0.861, respectively. These results show that there is a clear distinction between urine samples before and after training. It can be seen from the experiment that the main metabolites contributing to the differentiation of urine samples before and after training are lactic acid (LAC) and glycine (Gly), and n-trimethylamine oxide (TMAO) in urine increased significantly after training, while creatinine (CR) decreased.

Because the contents of lactic acid and creatinine changed dramatically after training, the integral values of these two metabolites were omitted, and further multivariate statistical analysis was carried out. It was found that the samples before and after training were significantly different.

The PCA, PLS-DA, and OPLS-DA sample score plots have cluster distribution between the two groups. The Q2 value of the OPLS-D model is 0.722, which is greater than 0.4. The arrangement experiment shows that the Q2 value of the rightmost is greater than that of all the left and R2X and R2Y are 0.436 and 0.85, respectively. These results show that there is a clear distinction between urine samples before and after training.

## 5. Conclusion

This paper presents a method of metabonomics study after exercise fatigue based on NMR. Through experiments, this method is used to explore the data comparison of urine components before and after athletes, so as to explore the physical status of athletes before and after sports. The experimental results show that Q2 value is greater than all Q2 values on the left and R2X and R2Y are 0.436 and 0.85, respectively. It also proves that the research method of metabonomics after exercise fatigue based on NMR can effectively prevent athletes' exercise fatigue.

## Figures and Tables

**Figure 1:** Flowchart of metabonomics experimental research.

**Figure 2:** Training contents and sampling flowchart of athletes in this study.

**Figure 3:** Metabolic diagram of the pro-phosphate system.

**Figure 4:** Energy supply of the glycolysis system.

**Figure 5:** Variation of running quantity of each quality around.

**Table 1:** List of heart rate changes of athletes in this study ($n=14,\bar{X}\pm \text{SD}$, times /min).

Basal heart rate	Training session average heart rate	Maximum heart rate in training session
48.4 ± 1.6	168 ± 2.9	202 ± 3.1

## Data Availability

The data used to support the findings of this study are available from the corresponding author upon request.
